The article "Reassortant between Human-Like H3N2 and Avian H5 Subtype Influenza A Viruses in Pigs: A Potential Public Health Risk" was published in 2010. Journal: PLoS One.

# Reassortant between Human-Like H3N2 and Avian H5 Subtype Influenza A Viruses in Pigs: A Potential Public Health Risk

**DOI:** 10.1371/journal.pone.0012591

**Published:** 2010-09-07

**Authors:** Yanlong Cong, Guangmei Wang, Zhenhong Guan, Shuang Chang, Quanpeng Zhang, Guilian Yang, Weili Wang, Qingfeng Meng, Weiming Ren, Chunfeng Wang, Zhuang Ding

**Affiliations:** 1 College of Animal Science and Veterinary Medicine, Jilin University, Changchun, Jilin, China; 2 Institute of Zoonoses, Jilin University, Changchun, Jilin, China; 3 College of Animal Science and Technology, Jilin Agricultural University, Changchun, Jilin, China; 4 Jilin Entry-Exit Inspection and Quarantine Bureau, Changchun, Jilin, China; Cairo University, Egypt

## Abstract

**Background:**

Human-like H3N2 influenza viruses have repeatedly been transmitted to domestic pigs in different regions of the world, but it is still uncertain whether any of these variants could become established in pig populations. The fact that different subtypes of influenza viruses have been detected in pigs makes them an ideal candidate for the genesis of a possible reassortant virus with both human and avian origins. However, the determination of whether pigs can act as a “mixing vessel” for a possible future pandemic virus is still pending an answer. This prompted us to gather the epidemiological information and investigate the genetic evolution of swine influenza viruses in Jilin, China.

**Methods:**

Nasopharyngeal swabs were collected from pigs with respiratory illness in Jilin province, China from July 2007 to October 2008. All samples were screened for influenza A viruses. Three H3N2 swine influenza virus isolates were analyzed genetically and phylogenetically.

**Results:**

Influenza surveillance of pigs in Jilin province, China revealed that H3N2 influenza viruses were regularly detected from domestic pigs during 2007 to 2008. Phylogenetic analysis revealed that two distinguishable groups of H3N2 influenza viruses were present in pigs: the wholly contemporary human-like H3N2 viruses (represented by the Moscow/10/99-like sublineage) and double-reassortant viruses containing genes from contemporary human H3N2 viruses and avian H5 viruses, both co-circulating in pig populations.

**Conclusions:**

The present study reports for the first time the coexistence of wholly human-like H3N2 viruses and double-reassortant viruses that have emerged in pigs in Jilin, China. It provides updated information on the role of pigs in interspecies transmission and genetic reassortment of influenza viruses.

## Introduction

The pig is considered to be an important host of influenza A viruses as it might be associated with the generation of human pandemic influenza strains [1]. Historically, two human pandemic viruses, H1N1 in 1918 and H3N2 in 1968, were almost simultaneously detected both in humans and pigs [2], [3]. Although the pandemic H3N2 virus was initially detected in humans and the full genome of the 1918 H1N1 pandemic virus was recently decoded [4], it is still unknown whether these viruses were first introduced into humans or into pigs before they became human pandemic strains.

The article "Reassortant between Human-Like H3N2 and Avian H5 Subtype Influenza A Viruses in Pigs: A Potential Public Health Risk" was published in 2010. Journal: PLoS One.

Currently, H1N1, H1N2 and H3N2 influenza subtype viruses co-circulate in pigs widely throughout the world. All of these viruses were the result of either interspecies transmission or reassortment events [5]–[7]. The Sydney-like H3N2 variants from pigs in the U.S.A. in 1998 were double and triple reassortants containing viral genes of human, swine and avian origin [8]. This highlights the complex and dynamic influenza ecology in pig populations.

Here we present the results of the genetic and phylogenetic characterization of swine H3N2 influenza viruses isolated from 2007 to 2008 in Jilin province of China. Genetic analysis showed that wholly contemporary human-like H3N2 viruses and double-reassortant viruses containing genes from contemporary human (PB2, PB1, PA, HA, NP, and NA) and avian H5 (M and NS) viruses were co-circulating in pig populations. This is the first description of an instance of reassortment between mammal H3N2 and avian H5 influenza viruses. The coexistence of entirely contemporary human-like viruses and double-reassortant viruses provides further evidence that pigs serve as intermediate hosts or mixing vessels. This emphasizes the importance of reinforcing swine influenza virus surveillance.

## Results

### HA1 amino acid analysis

To investigate all of the detailed genetic characteristics, we compared the deduced amino acid sequences of the hemagglutinin 1 (HA1) gene from the three swine H3N2 isolates against the representatives of five lineages (avian, European swine, earliest human, early human and contemporary human) available in GenBank. For the five lineages, the three H3N2 isolates showed a close relationship to HA1 genes from the contemporary human lineage with a sequence similarity of 94.8∼97.6% to Moscow/10/99, while there was 80.9∼87.2% similarity compared with the representatives of four other lineages (Dk/Hong Kong/7/75 (ABB88256.1), Sw/Italy/1461/96 (CAC40048.1), Hong Kong/1/68 (ACU79871.1), Port Chalmers/1/73 (AAC78096.1), and Victoria/3/75 (CAA24270.1)).

Analysis of amino acid variations of the proposed antigenic sites [9]–[11], receptor-binding sites [12], and potential glycosylation sites was conducted and variations are shown in Figure 1. The HA1 domain of HA, the major antigenic protein of influenza A viruses, contains all the antigenic sites of HA and is under continual immune-driven selection. For H3N2 viruses, the antigenic sites A∼E have been described [9]–[11]. All variations were accumulated at the antigenic sites A and B, while C, D and E were relatively conserved for the contemporary human-like H3N2 lineage. Concerning the three swine H3N2 isolates, two or four amino acid substitutions were observed at the major antigenic sites (A and B) of the HA1 molecule compared with Moscow/10/99, the representative for contemporary human lineage (Figure 1 and 2).

The article "Reassortant between Human-Like H3N2 and Avian H5 Subtype Influenza A Viruses in Pigs: A Potential Public Health Risk" was published in 2010. Journal: PLoS One.

**Figure 1:** Alignment of the HA1 amino acid sequences of three swine H3N2 influenza virus isolates and the representatives of five H3N2 lineages. The underlined residues represent the antigenic sites (lowercase letters indicate discrete antigenic sites), residues in green represent the potential glycosylation sites, and residues in yellow shade denote the receptor-binding sites.

**Figure 2:** Cartoon diagram representing the amino acid changes at the HA1 molecule of H3 subtype influenza viruses. RBD: receptor-binding domain. A, B and C: major antigenic sites at the HA molecules. Yellow color: conserved amino acids and red color: changed amino acids. (|) Sw/Jilin/5/07 vs. Moscow/10/99, (||) Sw/Jilin/19/07 vs. Moscow/10/99, (|||) Sw/Jilin/37/08 vs. Moscow/10/99.

Amino acids at the receptor-binding sites of the HA1 protein are associated with the differences in the receptor-binding specificity [13]. All of the H3N2 viruses had relatively conserved receptor-binding sites at Y98, G134, S136, W153, H183, Y195, and R224. Eight obvious mutations (A/S131T, T135G, H155T/Y, Q156K, K/Q158G, D190E, S193N, I/V194L) occurred between the contemporary human lineage and other lineages; these mutations were unique to the contemporary human lineage. Residues responsible for the sialic acid-α2,6-galactose (SAα2,6Gal) of H3N2 are L226 and S228 [14]. The viruses of avian lineage had Q at position 226, while the viruses of European swine, earliest human, and early human lineages had L, and the viruses of contemporary human lineage had I/V. The viruses of avian lineage had G at position 228, with other four lineages being S. In this study, all of the swine H3N2 isolates contained V instead of L at position 226.

It has been considered that carbohydrate side chains might affect receptor-binding capacity and antigenicity [11], [15], [16]. Analysis of potential glycosylation sites in the HAs of the three H3N2 isolates revealed eight common sites (N8, 22, 38, 63, 122, 133, 165 and 285, respectively) with the NXT/S motif (in which X may be any amino acid except aspartic acid and proline). Furthermore, as shown in Figure 1, both Sw/Jilin/5/07 and Sw/Jilin/19/07 possessed an additional glycosylation site at position 126, and Sw/Jilin/5/07 acquired another one at position 246.

The article "Reassortant between Human-Like H3N2 and Avian H5 Subtype Influenza A Viruses in Pigs: A Potential Public Health Risk" was published in 2010. Journal: PLoS One.

### Phylogenetic analysis

Phylogenetic analysis and identification of antigenically different strains are necessary to monitor the evolution of influenza virus. The phylogenetic relationships among swine H3N2 viruses prevalent in Jilin province compared to the selected reference strains available in the GenBank were estimated from the nucleotide sequences of each viral gene. The phylograms for all genes are shown in Figures 3a∼3h.

**Figure 3:** Phylogenetic trees of the eight gene segments of the influenza viruses. The tree was created by the neighbor-joining method and bootstrapped with 1,000 replicates. The bootstrap numbers are given for each node. Only bootstrap values above 80 are shown. Viruses isolated in the present study are in bold. Abbreviations used in virus designations are as follows: Ck, chicken; Dk, duck; Sw, swine; Tk, turkey.

Phylogenetic analysis of H3 HAs showed that H3N2 viruses could be segregated into five distinct lineages, including avian strains, European swine strains, earliest human strains, early human strains, and contemporary human strains (Figure 3a). The swine viruses of earliest human lineage seemed to be derived from the human strain A/Hong Kong/1/68. The early-human-derived swine viruses were closely related to A/Victoria/75-like viruses. The swine viruses of European swine lineage were probably derived from European H3N2 swine influenza viruses, for which the HA genes originated from A/Victoria/3/75. The contemporary human lineage included three sublineages (represented by Sydney/97-like, New York/99-like and Moscow/99-like viruses). The HAs of the three swine H3N2 virus isolates tested in this study clustered into the Moscow/99-like virus sublineage.

The phylogeny of the NA and internal genes of H3N2 viruses paralleled to that of the HA genes, in which five different lineages were defined. The NA, PB2, PB1, PA, and NP genes of the three isolates in this study belonged to the contemporary human lineage. Additionally, in the NA tree, Sw/Jilin/37/08 was equally closely related to the early and contemporary H3 strains as well as an intermediate swine virus between the early lineage and the contemporary human lineage. In the M and NS trees, Sw/Jilin/5/07 and Sw/Jilin/19/07 still clustered in the contemporary human lineage, whereas Sw/Jilin/37/08 was incorporated into the avian lineage (Figures 3b∼3h).

The results of the published data in GenBank revealed that in recent years H3N2 influenza viruses were cocirculating with H5 influenza viruses, raising the possibility of genetic exchange between these viruses. The evolutionary trees revealed that the M gene of Sw/Jilin/37/08 formed a sublineage with H5N3 viruses (A/Dk/Altai/1285/1991, A/Dk/Primorie/2633/2001, A/Anasplatyrhynchos/Altai/1285/1991, and A/Migratory Dk/Jiangxi/13487/2005 (Figure 3g)). The NS gene of Sw/Jilin/37/08 had a close relationship with A/Mallard/Italy/4223-2/2006 (H5N2) and A/Dk/Primorie/2633/2001 (H5N3) (Figure 3h).

The article "Reassortant between Human-Like H3N2 and Avian H5 Subtype Influenza A Viruses in Pigs: A Potential Public Health Risk" was published in 2010. Journal: PLoS One.

## Discussion

The rapid evolution of influenza viruses occurs both clonally and non-clonally through a variety of genetic mechanisms and selection pressure. Three mechanisms on the non-clonal evolution of influenza viruses have been proposed: (i) relatively frequent reassortment among gene segments of multiple host types, (ii) possibly but rarely non-homologous recombination, in which short regions of sequence are transferred among different segments, and (iii) controversial and extremely rare homologous recombination within segments [17]. Reassortment, therefore, plays an important role in the non-clonal evolution of the influenza viruses.

Infection of pigs with H1, H3, H5 and H9 subtype influenza viruses has occurred frequently on multiple occasions [5], [18]–[23]. As pigs can serve as intermediate hosts or mixing vessels for the reassortment of human and avian influenza viruses, swine influenza infections have been the focus of increasing attention. It often appeared that multiple reassortments occurred among the same subtype or different subtypes of human, swine and avian viruses in pig populations. The best examples are the swine H1N2 isolates and the pandemic novel H1N1 influenza virus that emerged in the human population. Peiris et al [24] were the first to confirm that cocirculation of contemporary human H3N2 viruses and avian H9N2 in pigs had occurred in southeastern China. Xu et al [25] reported that the avian H9N2 viruses caused pig disease and death in clinics, and deduced that it probably originated from a reassortant of avian H5 influenza virus and H9N2 viruses. All of these situations indicated that the cocirculation of H1, H3, H5 and H9 viruses in pigs would provide an opportunity for genetic reassortment, leading to the emergence of viruses with pandemic potential. Avian influenza viruses, especially when avian H5 subtype viruses reassorted with suitable surface glycoproteins, can infect humans [26]. Yu et al [27] described the coexistence of wholly human-like H3N2 viruses, double-reassortant and triple-reassortant H3N2 viruses in pigs in China from 1970 to 2006. However, reassortment was not found between mammal H3N2 viruses and avian H5 viruses. From July 2007 to October 2008, we collected 279 nasopharyngeal swabs from pigs diagnosed with respiratory tract illness on different pig farms in Jilin province. The H3N2 influenza virus infections in the pigs were diagnosed by virus isolation. The results showed that one Moscow/10/99-like reassortant isolate, A/swine/Jilin/37/2008, contained avian H5-like M and NS genes, suggesting that after introduction to pigs, avian H5 viruses further reassorted with contemporary human-like H3N2 viruses. To our knowledge, such reassortment between mammal H3N2 viruses and avian H5 viruses has not been described in existing publications.

The article "Reassortant between Human-Like H3N2 and Avian H5 Subtype Influenza A Viruses in Pigs: A Potential Public Health Risk" was published in 2010. Journal: PLoS One.

A comparison of the amino acid sequences of the HA1 region of our isolates with the representatives of avian lineage (Dk/Hong Kong/7/75), European swine lineage (Sw/Italy/1461/96), earliest human lineage (Hong Kong/1/68), early human lineage (Victoria/3/75 and Port Chalmers/1/73), and contemporary human lineage (Sydney/5/97, New York/185/99, and Moscow/10/99) showed that the three H3N2 swine isolates were more closely related to Moscow/10/99 (94.8∼97.6% amino acid similarity), indicating that the HAs of them seemed to be derived from those of the contemporary human lineage. Phylogenetic analysis of the HAs also suggested that the three H3N2 isolates had been introduced into pigs at several points in time from the human side.

The comparison of antigenic sites of HA1 regions revealed evolution by antigenic drift of their HA genes. Codons under positive selection were associated with antigenic site A and B [28]. Sw/Jilin/19/07 had two variations at the antigenic sites A and B, while Sw/Jilin/5/07 and Sw/Jilin/37/08 accumulated four variations at the antigenic sites A and B. The gradual mutations of HA might generate new antigenic strains. Wilson and Cox [29] proposed that a drift variant with ≥4 amino acid changes at ≥2 out of 5 antigenic sites would be of epidemiologic importance. It has been also observed that new antigenic variations are created either when ≥2 variations occur in antigenic sites or when one variation occurs in an antigenic site and one in a sialic acid receptor-binding site [30].

Although the molecular basis of host-range restrictions is not completely defined, the compatibility between the HA protein of the virus and its corresponding receptor, sialic acid, on the host cell is thought to contribute in part to the infection of the virus in a specific host [31], [32]. Pigs, unlike humans, seem to be readily infected by most, if not all, mammalian and avian influenza viruses. The susceptibility of pigs to both mammalian and avian viruses is due to the presence of receptors for both lineages of virus in the pig trachea [33]. For H3N2 viruses, residues 226 and 228 on the receptor-binding domain of the HA1 molecule were shown to play a critical role in determining receptor specificity [14], [34], [35]. The three H3N2 isolates possess V226 and S228, which are the same as those of both turkey and swine triple reassortants. While L/I226 and S228 are usually expressed in human viruses [36], Q226 and G228 are usually found in avian viruses [14]. V, L and I are neutral non-polar amino acids, and substitutions between them most likely maintain the hydrophobic interactions and the proper 3D conformation at the binding domain [37].

The article "Reassortant between Human-Like H3N2 and Avian H5 Subtype Influenza A Viruses in Pigs: A Potential Public Health Risk" was published in 2010. Journal: PLoS One.

Carbohydrate side chains are important for the structure and stability of glycoproteins [38], [39]. Changes in carbohydrate side chains are an important mechanism in the structural variation underlying antigenic drift. In this study, the three swine H3N2 isolates had eight to ten glycosylation sites, although all of them may not be used. Of these sites, positions 122, 133, and 246 were unique to the contemporary human lineage. In addition, the lineages of European swine, earliest human, early human, and contemporary human had more glycosylation sites than the avian lineage. The addition of new carbohydrate side chains to HA may have provided the viruses with the ability to evade antibody pressure by changing the antigenicity and by having an increased ability to prevail. For instance, human virus variants which cocirculated in the epidemic area with a higher number of glycosylation sites appeared to prevail at the end of the outbreak [40]. Conclusively, molecular analysis of the hemagglutinin gene showed that the 2007–2008 H3N2 influenza viruses circulating in swine populations in Jilin province accumulate variations at the antigenic sites A and B, receptor-binding sites, as well as glycosylation sites.

Phylogenies of the whole genome of the swine H3N2 influenza viruses in Jilin province, China during 2007 to 2008 provided evidence of the persistence of both the contemporary human lineage and the avian lineage in pig populations. These results also revealed multiple interspecies transmissions of influenza viruses from human and avian to pig and subsequent reassortment events, particularly together with the participation of internal genes from the avian H5 lineage in this region. This is the first report on reassortment between mammal H3N2 and avian H5 viruses.

Experimental infection suggested that introduction of certain H5 viral segments into circulating human H3N2 viruses may increase their virulence for mice and perhaps other mammalian species [41]. Further research is needed to determine whether Sw/Jilin/37/08 has higher virulence than Sw/Jilin/5/07 and Sw/Jilin/19/07. The principal evolutionary mechanism of influenza virus is by antigenic drift, creating small progressive antigenic changes in the hemagglutinin and neuraminidase surface antigens [42]. However, genetic reassortment readily occurs between influenza viruses and may also contribute to the evolution of new strains. Therefore Sw/Jilin/37/08 may represent a potential threat in the emergence of new human viruses.

The article "Reassortant between Human-Like H3N2 and Avian H5 Subtype Influenza A Viruses in Pigs: A Potential Public Health Risk" was published in 2010. Journal: PLoS One.

There have been numerous descriptions of human infection with swine influenza viruses [5]. The swine populations have become a reservoir of a much more diverse array of influenza viruses. The replicative gene constellation of H3N2 viruses has the capacity to reassort among avian, swine and human viruses. This means that activity in swine virus reservoirs is of concern for human health. The above study provides additional evidence for continuing interspecies transmission and reassortment events occurring in pigs, which naturally increased the possibility of pigs as an important host for the emergence of novel reassortants with genes adapted for replication in pigs or even humans. The coexistence of reassortant viruses, especially reassortants of H3 and H5 viruses, emphasizes that genetic reassortment is an important factor in the evolution of H3N2 viruses and a formal surveillance system is needed for swine and avian influenza. It is only through such a system that cross-interspecies transmission and novel reassortment events will be identified in a timely fashion.

## Materials and Methods

### Viruses

A total of 279 nasopharyngeal swabs were collected in Jilin province, China from July 2007 to October 2008. The initial isolation of the viruses was performed in Madin-Darby canine kidney (MDCK) cells. The viruses were grown in Eagle minimal essential medium (GIBCO/BRL) supplemented with 5% fetal bovine serum (GIBCO/BRL), penicillin-streptomycin (GIBCO/BRL), amphotericin B (Fungizone; GIBCO/BRL) and tolylsulfonyl phenylalanyl chloromethyl ketone-treated trypsin (1 µg/ml; Worthington Biochemical Corporation, Lakewood, N.J.). Subtype identification of these viruses were determined by standard hemagglutination inhibition tests and neuraminidase inhibition tests with a panel of reference antisera recommended by the World Health Organization (http://www.who.Int/csr/resources/publications/en/#influenza). Viral fluids were harvested for MDCK-passaged viruses and used as stock for sequence analysis. The three H3N2 virus isolates obtained in this study were named as follows: A/swine/Jilin/5/2007 (Sw/Jilin/5/07), A/swine/Jilin/19/2007 (Sw/Jilin/19/07), and A/swine/Jilin/37/2008 (Sw/Jilin/37/08).

### Gene sequencing and phylogenetic analysis

Viral RNA was extracted using Trizol reagents (GIBCO/BRL) and reverse transcription was performed using oligonucleotide influenza universal primer Uni12: 5′-AGC AAA AGC AGG-3′ [43]. After reverse transcription, PCR was done as described by Shu [44] using primers (Table 1) specific for each of the eight RNA segments. PCR products were purified with the QIA quick PCR purification kit (Qiagen). The purified PCR products were then partially sequenced using an Amersham ET Dye terminator kit and analyzed with an ABI 3730 DNA sequencer (Perkin-Elmer Appllied Biosystems, Foster City, CA, USA).

The article "Reassortant between Human-Like H3N2 and Avian H5 Subtype Influenza A Viruses in Pigs: A Potential Public Health Risk" was published in 2010. Journal: PLoS One.

**Table 1:** The primer sequences used for PCR amplification of H3N2 influenza virus genes.

Gene	Forward primer 5′→3′	Reverse primer 5′→3′	Expected size (bp)
**PB2**	GCTGATAGTGAGTGGAAGAGACGAACA	AGTAGAAAAAGGTCGTTTTTAAACTATTC	1166
**PB1**	TGCGAGCTGACTGATTCAATCTGGATA	AGTAGAAACAAGGCATTTTTTCATGAA	2321
**PA**	TGCGAGCTGACTGATTCAATCTGGATA	AGTAGAAACAAGGTACTTTTTTGGACA	967
**HA**	ATGAAGACTATCATTGCTTTGAGCTAC	TCAAATGCAAATGTTGCACCTAATG	1701
**NP**	AGCAAAAGCAGGGTAGATAATCACTCA	AGTAGAAACAAGGGTATTTTTCTTTAA	1565
**NA**	AGCAAAAGCAGGAGTAAAGATGAAT	AAGCTTATATAGGCATGAGATTGAGG	1433
**M**	ATATTGAAAGATGAGCCTTCTAACCG	ACTCCAACTCTATGCTGACAAAATGAC	990
**NS**	AGCAAAAGCAGGGTGACAAAGACATAA	AGTAGAAACAAGGGTGTTTTTTATTAT	890

Assembly of sequences, translation of nucleotide sequences into protein sequences, and initial multiple sequence alignments were performed with the Clustal V method using MegAlign software version 1.03 (SNAStar Inc., Madison, WI).

The reference strains selected for phylogenetic analysis are based on the following criteria: 1. Using a blast search (http://blast.ncbi.nlm.nih.gov/Blast.cgi), the most genetically closest segment sequence is selected. 2. The selected strains are well-characterized phylogenetically, so that they can represent their lineage and host origin, such as avian, pig or human. 3. The general topology of the phylogenetic tree constructed using the selected reference strains is consistent with previously well-recognized evolutionary analysis. Bootstrap support for tree topologies was accomplished using the Neighbor-joining (NJ) methods implemented in MEGA 4.0 with 1,000 iterations [45]. Genetic distances based on NJ phylogenetic trees were calculated applying Kimura's two-parameter method. In this study, the nucleotide sequences used for the phylogenetic analysis are as follows: PB2 1185-2306, PB1 64-2241, PA 1266-1579, HA 78-1064, NP 46-1504, NA 89-1399, M 35-990, and NS 27-822.

### Molecular graphic visualization

Amino acid changes at the five antigenic sites (A∼E) [9]–[11] of the HA1 molecule were determined by amino acid sequence alignment using the MegAlign program. Changes at the major antigenic sites (A, B and C) of the HA monomer were located using PyMOL software (v0.99) (DeLano Scientific LLC, South San Francisco, California, U.S.A.) based on the HA structure of the H5 subtype influenza virus, A/duck/Singapore/3/97 [46], (1JSM) downloaded from the Protein Data Bank website (http://www.rcsb.org/pdb/home/home.do). The H5 structure was used because it is available as a monomer structure and it would be clearer to visualize the amino acid changes on it than the H3 structure, which is only available as a trimer structure.

The article "Reassortant between Human-Like H3N2 and Avian H5 Subtype Influenza A Viruses in Pigs: A Potential Public Health Risk" was published in 2010. Journal: PLoS One.

### Nucleotide sequence accession numbers

The nucleotide sequences for all H3N2 influenza virus isolates analyzed in this study are available from GenBank under accession numbers GU215015 to GU215038 (Table 2).

**Table 2:** The accession numbers of protein and nucleotide acid of swine H3N2 influenza viruses.

	A/swine/Jilin/5/2007				A/swine/Jilin/19/2007				A/swine/Jilin/37/2008			
	Protein		Nucleotide acid		Protein		Nucleotide acid		Protein		Nucleotide acid	
	Accession	Length (aa)	Accession	Length(bp)	Accession	Length(aa)	Accession	Length(bp)	Accession	Length(aa)	Accession	Length(bp)
**PB2**	ACZ53952	373	GU215015	1121	ACZ53963	373	GU215023	1121	ACZ53974	373	GU215031	1121
**PB1**	ACZ53953	757	GU215016	2317	ACZ53964	757	GU215024	2317	ACZ53975	757	GU215032	2317
**PA**	ACZ53955	302	GU215017	930	ACZ53966	302	GU215025	930	ACZ53977	302	GU215033	930
**HA**	ACZ53956	566	GU215018	1701	ACZ53967	566	GU215026	1701	ACZ53978	566	GU215034	1701
**NP**	ACZ53957	498	GU215019	1541	ACZ53968	498	GU215027	1541	ACZ53979	498	GU215035	1541
**NA**	ACZ53958	469	GU215020	1414	ACZ53969	469	GU215028	1414	ACZ53980	469	GU215036	1414
**M1**	ACZ53959	249	GU215021	957	ACZ53970	249	GU215029	957	ACZ53981	249	GU215037	957
**NS1**	ACZ53961	230	GU215022	890	ACZ53972	230	GU215030	890	ACZ53983	230	GU215038	890
